RETRACTED

# Butylphthalide Inhibits TLR4/NF-*κ*B Pathway by Upregulation of miR-21 to Have the Neuroprotective Effect

**DOI:** 10.1155/2022/4687349

**Published:** 2022-01-07

**Authors:** Lan Zhan, Yu Pang, Hao Jiang, Shicun Zhang, Hongwei Jin, Jing Chen, Cuiying Jia, Hongyan Guo, Zhuang Mu

**Affiliations:** ^1^Department of Neurology, The Second Affiliated Hospital of Qiqihar Medical University, Qiqihar 161000, China; ^2^Department of Clinical Laboratory, The Second Affiliated Hospital of Qiqihar Medical University, Qiqihar 161000, China; ^3^Department of Biochemistry Teaching and Research, Qiqihar Medical University, Qiqihar 161000, China; ^4^Department of Neurosurgery, The First Hospital of Qiqihar City, Qiqihar 161000, China

## Abstract

Stroke is a disease with the highest incidence rate and the highest mortality rate in the world. The study aims to verify the neuroprotective effect of Butylphthalide. The mice were divided into sham group, MCAO group, and MCAO + Butylphthalide-treated group. The mice in MCAO + Butylphthalide-treated group were administered with 70 mg/kg Butylphthalide injection intraperitoneally after cerebral ischemia-reperfusion. The normal saline with the same volume was administered intraperitoneally for the mice in the MCAO group and sham group. The levels of miR-21 in brain tissue and cells were detected by qPCR. The OGD/R injury model of Neuro2A cells was used to simulate the hypoxic-ischemic environment of neurons in vitro. The proliferation rate of Neuro2A cells was detected with CCK-8. The production of ROS was detected with DCFH-DA. Compared with the mice in MCAO group, a decrease (*P* < 0.01) was observed in the functional neurologic impairment scoring, cerebral infarction volume, and brain loss volume in the mice treated with MCAO + Butylphthalide, but an increase (*P* < 0.01) was observed in the level of miR-21, which was positively correlated with functional neurologic impairment scoring (*r* = −0.8933, *P* < 0.001). MTT assay showed that the cell viability of OGD/R + Butylphthalide group was significantly higher than that of other groups (*P* < 0.001), and the activity of ROS was significantly decreased (*P* < 0.001). The WB results showed that, compared with OGD/R + miR-NC and control groups, the ratio of Bcl-2/Bax in OGD/R + Butylphthalide group and OGD/R + miR-21 mimics group was significantly higher (*P* < 0.05), while the ratio of caspase-3/GAPDH was significantly lower (*P* < 0.05). In conclusion, Butylphthalide has neuroprotective effect on the mouse model of MCAO. It may upregulate the level of miR-21 to inhibit neuronal apoptosis and ROS production and improve the proliferation activity. The specific mechanism may lie in inhibiting TLR4/NF-*κ*B pathway.

RETRACTED

## 1. Introduction

Stroke is a disease with the highest incidence rate and the highest mortality rate in the world [1]. Among all the cases, ischemic stroke accounts for about 87%. Most of the patients have the serious functional neurologic disorder, which brings serious economic burden to their families and society [2]. Dl-3-n-Butylphthalide (NBP) (chemical formula: C12H14O2, molecular weight: 190.24) is a synthetic compound based on l-3-n-Butylphthalide which is isolated from celery seed. Many clinical studies have shown that NBP is a safe and effective treatment for ischemic stroke. It not only relieves the symptoms of ischemic stroke but also contributes to long-term rehabilitation [3–5].

NBP has shown a protective effect on ischemic stroke in various animal models [6–12]. However, its specific mechanism is not defined. Its protective effect may be related to the increase of local blood flow [6, 13], and the decrease of brain edema and blood-brain barrier damage [8] as well as fewer chances of thrombosis [14, 15]. In addition, studies have shown that NBP can reconstruct microcirculation and reduce the content of arachidonic acid (AA), inhibit human platelet phosphodiesterase and increase the level of 3,5-cyclic adenosine monophosphate in platelets, and increase the content of nitric oxide (NO) and PGI2 in cerebral vascular endothelial cells, improving arterial microcirculation [7]. NBP can increase the activities of Na + - K + ATPase and Ca2+-ATPase in mitochondrial membrane, improve the decrease of neuron mitochondria complex IV activity induced by hypoglycemia and hypoxia, and increase the activities of SOD and glutathione peroxidase (GSH-Px) in mitochondria. It can also decrease the release of cytochrome c and increase the activity of cytochrome c oxidase in mouse cells and inhibit caspase-dependent apoptosis. According to some other studies, NBP can inhibit ROS production by inhibiting nicotinamide adenine dinucleotide (NADH). Therefore, it can improve energy metabolism [16], reduce oxidative damage [17], prevent inflammatory reaction [18], and reduce neuronal apoptosis [19, 20].

Our previous study found that the level of miR-21 in the peripheral blood of ischemic stroke patients treated with Butylphthalide was increased. According to Jiansuo Zhou et al., the level of miR-21 in the plasma of patients with acute cerebral infarction was lower than that of the control group. Studies have confirmed the neuroprotective effect of miR-21 in cerebral ischemia-reperfusion injury and pointed out that MAP2K3 pathway can be used as the therapeutic target [21]. In addition, overexpression of miR-21 can prevent renal ischemic injury [22], which indicates that the level of miR-21 has a protective effect against ischemic diseases. Studies have shown that miR-21 is related to nerve repair and vascular protection after stroke. According to Buller et al.‘s in vivo and in vitro experimental studies, the level of miR-21 was significantly increased after ischemic stroke, inhibiting neuronal cell death by reducing Fas ligand (FasL) *G* (an important cell death-inducing ligand) [23]. miR-21 can participate in vascular remodeling by regulating VSMCs apoptosis and phenotype transformation and play an important role in neointimal formation in the induction model of intimal injury [21, 24]. TLR4/NF-*κ*B pathway plays an important role in ischemia-reperfusion injury. The overexpression of miR-21 can effectively inhibit TLR4/NF-*κ*B pathway, reducing the level of cardiomyocyte apoptosis and the release of inflammatory factors of mice [25]. Other studies have shown that miR-21 can protect against ischemic injury through PDCD4/NF-*κ*B pathway [26]. These results suggest that miR-21 can affect the neurovascular unit remodeling by regulating neuronal apoptosis and angiogenesis. The protective mechanism of Butylphthalide on cerebral ischemia may be achieved by miR-21 regulation. This study aims to clarify the neuroprotective mechanism of Butylphthalide through miR-21.

RETRACTED

## 2. Methods

### 2.1. Animal Model

Male C57BL/6 mice aged 8–10 weeks were purchased from Shanghai Lab Animal Research Center and fed in SPF animal room. The mice were divided into three groups: sham operation group, MCAO group, and MCAO + Butylphthalide-treated group, with 5 mice in each group. Mice were anesthetized with ketamine (100 mg/kg) and xylazine (10 mg/kg). After midline skin incision, the left common carotid artery was exposed and electrocoagulation was performed on its branches. Two centimeters were slowly pushed from the external carotid artery bifurcation to the internal carotid artery, and a 6–0 round nylon suture was used. After 60 minutes of proximal MCA obstruction, blood flow was restored after the removal of the suture. In the sham group, the carotid artery was exposed without middle cerebral artery ligation. The mice in MCAO + Butylphthalide-treated group were administered with 70 mg/kg Butylphthalide injection intraperitoneally after cerebral ischemia-reperfusion once a day. The normal saline with the same volume was administered intraperitoneally for the mice in MCAO group and sham group. After a 60-minute MCAO, blood perfusion was restored for 72 hours. During the operation, the rectal temperature was controlled at 37.0 ± 0.5°C with heating pad. With ischemic injury, mice were placed in a ventilated incubator at 24.0 ± 0.5°C. After 72 hours of reperfusion, all mice had the functional neurologic impairment scoring, and then the animals were killed and their brains were taken out quickly to confirm the infarct. According to Longa's 5-grade scoring standard, the functional neurologic impairment was assessed as “no symptoms of functional neurologic impairment [0],” “the contralateral forepaw of cerebral ischemia could not be fully extended [1],” “turning to the opposite side [2],” “dumping to the opposite side [3],” “involuntary walking and unconsciousness [4]”, and “death [5]”. All procedures for the use of laboratory animals were approved by the animal ethics committee of the Second Affiliated Hospital of Qiqihar Medical University. The protocol fully complies with the *Guide for Care and Use of Laboratory Animals of National Institutes of Health* (NIH publication 85–23, revised in 1996).

RETRACTED

### 2.2. Calculation of Infarct Volume and Brain Loss Volume

The infarct volume was measured with 2,3,5-triphenyltetrazolium chloride (TTC) [27]. The brain was cut into four coronal sections with the thickness of 0.2–0.3 cm. The slices were immersed in 2% 2,3,5-triphenyltetrazolium chloride (TTC) for 30 minutes at 37°C, and the images were scanned into a computer to be measured with imaging analysis software (Image *J*, 1.52a). The infarct volume (cm^3^) of each slice was equal to the infarct area (cm^2^) multiplied by the slice thickness (0.2 cm or 0.3 cm). The total infarct volume of each brain was then calculated by summing the infarct volumes of all slices. In order to minimize the effect of edema on the accuracy of infarct volume measurement, the final infarct volume was corrected with a coefficient equal to the ratio of nonischemic hemisphere volume to the ischemic one. Hematoxylin and Eosin (H&E) staining was performed to detect brain loss. Brain loss was measured by subtracting the nonlesion area of the ipsilateral hemisphere from the contralateral hemisphere. The volume of tissue loss was calculated with the lesion area of six parts and analyzed with Image *J* (1.52a).

### 2.3. Cell Culture and Oxygen-Glucose Deprivation/Reoxygenation (OGD/R) Cell Model

Neuro2A was purchased from American Type Culture Collection (ATCC, Shanghai, China). Cells were cultured under normal conditions (95% air, 5% CO2) with conventional high-glucose DMEM containing 10% FBS (Gibco) in an incubator at 37°C. As the density of the cells grew to 50%, the old medium was replaced with Hanks Balanced Salt (HBSS; glucose concentration = 0 mg/dL) and the medium was transferred to the anoxic chamber (95% nitrogen and 5% CO_2_) for 3 hours. At the end of OGD phase, the medium was replaced with the original complete medium and cultured under normal conditions for 24-hour reoxygenation. Cells without OGD/R treatment were used as a control. After OGD/R, the medium in Butylphthalide-treated group was replaced with a complete medium containing 10 *μ*m Butylphthalide. All chemicals/drugs have been sterilized.

RETRACTED

### 2.4. Cell Transfection

MiR-21 mimics, miR-21 inhibitor, and negative control (miR-NC or anti-miR-NC) were purchased from GenePharma. When the density of Neuro2A cells grew to 70%, Lipofectamine 2000 Reagent (Invitrogen, USA) was used to transfect the cells with miR-211 mimics or inhibitor or negative control according to the operating procedure of the manufacturer, and the final concentration was 50 nM. The cells were harvested 24 hours after transfection for further study, and then the above cells were placed in OGD/R.

### 2.5. Real-Time Fluorescence Quantitative PCR

Total RNA and miRNA were extracted from cerebral infarction tissues and Neuro2A cells with miRNeasy Mini Kit (Qiagen, Germany). TaqMan microRNA Reverse Transcription Kit (California, Applied Biosystems) was used to obtain cDNA, and TaqMan miRNA Kit (Applied Biosystems) was used for qRT-PCR. The reaction procedure was as follows: initial denaturation: 95°C, 30 sec; circular reaction: 60°C, 20 sec, 40 cycles. U6 small nuclear RNA (U6 snRNA) was used as a standardized endogenous control. SYBR Green mix (TaqMan) was used to perform qRT-PCR on 7900HT rapid real-time PCR system (Applied Biosystems). U6 was used as the internal control and the changes of miRNA level were quantified by 2-ΔΔCT. The primer sequence is shown in Table 1.

### 2.6. MTT Assay

Neuro2a cells were seeded into a 96-well plate at a density of 10^5. After overnight culture, transfection or Butylphthalide treatment was given according to the requirements of each group with MTT cell proliferation and cytotoxicity detection kit (Beyotime). Then 10 *μ*L MTT solution was added to each well and they were continued to be incubated for 4 hours in the cell incubator. 100 *μ*L formazan solution was added into each well. After mixing, they were continued to be incubated in the cell incubator. The incubation did not stop until the formazan was completely dissolved under the ordinary optical microscope. Generally, after incubation at 37°C for 3–4 hours, all purple crystals will dissolve. The absorbance value was measured at 570 nm and observed under 20x optical microscope.

### 2.7. WB Experiment

The cells were sonicated for 1 minute in the precooled RIPA lysate (Beyotime) and centrifuged at 12,000 g for 10 minutes at 4°C and the supernatant was stored at −80°C. The protein concentration in the sample was determined with BCA Protein Assay Kit (Beyotime). Electrophoretic separation was performed for the extracted protein with 10% SDS-polyacrylamide gel and the protein was transferred to PVDF (Millipore, Bedford, MA, USA). The membrane was sealed in TBST buffer containing 5% skim milk for 1 hour and then incubated overnight at 4°C with the following primary antibodies: anti-mouse-p-tlr4 (Santa Cruz, 1 : 1000), anti-mouse TLR4 (CST, 1 : 1000), anti-mouse-p-nf-*κ* B (Santa Cruz, 1 : 1000), anti-mouse-NF-*κ* B (Santa Cruz, 1 : 1000), anti-mouse-casepse3 (abcam,1 : 1000), anti-mouse-Bax (abcam,1 : 1000), anti-mouse-Bcl-2 (abcam,1 : 1000), and anti-mouse-GAPDH (Santa Cruz, 1 : 1000). Then the membrane was washed with TBST and incubated with horse radish peroxidase labeled goat anti-rabbit IgG (Beyotime, A0216, 1 : 5000) for 1 hour at room temperature. Enhanced chemiluminescence detection system (Bio-Rad, Hercules, CA, USA) was used to detect protein bands, and Image Lab software (Bio-Rad) was used to quantify protein bands.

RETRACTED

### 2.8. Determination of Intracellular ROS

The cultured cells were digested with 0.04% Trypsin pancreatin and centrifuged at 1000 rpm for 5 minutes. DCFH-DA was diluted with serum-free medium at the ratio of 1 : 1000 through reactive oxygen species detection kit (Beyotime) to make the final concentration of 10 *μ*mol/L. The collected cells were suspended in diluted DCFH-DA and incubated for 20 minutes in the cell incubator at 37°C. The solution was mixed every 3–5 minutes to make the probe fully in contact with the cell. The cells were washed three times with serum-free cell culture medium to remove DCFH-DA from the cells. The production of ROS was detected with flow cytometry and quantified with CellQuest.

### 2.9. Statistical Analysis

SPSS 22.0 was used for statistical analysis. All experimental results were expressed as mean ± standard deviation. The difference of quantitative data between the two groups was compared with unpaired *t*-test. The quantitative data among multiple groups was analyzed with ANOVA. Bonferroni method was used for pairwise comparison between the two groups. *P* < 0.05 was considered as significant difference.

## 3. Results

### 3.1. Butylphthalide Improves Neurological Function Score and Reduces Cerebral Infarction Area in the Mouse Model of MCAO

In order to clarify the neuroprotective effect of Butylphthalide on ischemic stroke, the mouse model of MCAO was established. On the day of cerebral ischemia-reperfusion, 70 mg/kg Butylphthalide injection was administered intraperitoneally. The neurological function score and infarct area of the mice in MCAO group and MCAO + Butylphthalide-treated group were compared after 3-day administration in a row. It was found that the functional neurologic impairment score of the mice in the MCAO + Butylphthalide-treated group was significantly lower than that in MCAO group (Figure 1(a), *P* < 0.01). According to the calculated infarct size and brain loss volume, it was found that the infarct volume and brain loss volume of the mice in the MCAO + Butylphthalide-treated group were significantly lower than those in MCAO group (Figures 1(b) and 1(c); *P* < 0.05; *P* < 0.01). The level of miR-21 in infarcted brain tissue was further explored and it was found that the level of miR-21 of the mice in MCAO group was significantly lower than that in sham group (*P* < 0.001), while the level of miR-21 of the mice in Butylphthalide-treated group was significantly higher than that in MCAO group (*P* < 0.01), and there was no statistical difference between MCAO group and sham group (Figure 1(d)). According to the correlation analysis of neurological function score and miR-21 level, it was found that there was a negative correlation between them (Figure 1(e), *r* = −0.8933, *P* < 0.001).

RETRACTED

### 3.2. Butylphthalide and miR-21 Mimics Inhibit the OGD/R Injury of Neuro2A Cells

In order to further study the neuroprotective effect of Butylphthalide after ischemic stroke through miR-21, the OGD/R injury model of Neuro2A was established. The mice in OGD/R + Butylphthalide group were administered with 10 *μ*m Butylphthalide 24 hours after OGD/R treatment. For the mice in the OGD/R + Butylphthalide + miR-21 inhibitor group, they were administered with Butylphthalide and miR-21 inhibitor transfection was performed simultaneously after OGD/R injury occurred. As shown in Figure 2(a), the level of miR-21 in Neuro2A cells in OGD/R + Butylphthalide-treated group was significantly higher than that in OGD/R + miR-21NC group and control groups (*P* < 0.0001). However, after transfection of miR-21 inhibitor at the same time, the level of miR-21 did not increase significantly, but there was a significant decrease compared with that of OGD/R + Butylphthalide group (*P* < 0.001), and there was no significant difference with the control group. MTT assay showed that the cell viability in OGD/R + Butylphthalide group was significantly higher than that of other groups, while the cell viability in OGD/R + Butylphthalide + miR-21 inhibitor group was significantly lower than that in OGD/R + Butylphthalide group (*P* < 0.001); there was no significant difference in cell viability of OGD/R injury compared with that of the control group, and the cell viability in OGD/R + miR-NC group was the lowest (Figure 2(b)). The results of reactive oxygen species (ROS) measurement showed that the ROS activity in OGD/R + Butylphthalide group was significantly lower than that of OGD/R + Butylphthalide + miR-21 inhibitor group (*P* < 0.001), while the ROS activity in OGD/R + Butylphthalide + miR-21 inhibitor group was similar to that in OGD/R + miR-NC group, and the difference was not statistically significant (Figure 2(c)). These results suggested that Butylphthalide has neuroprotective effect through miR-21.

RETRACTED

### 3.3. Butylphthalide and miR-21 Mimics Inhibit the OGD/R Apoptosis of Neuro2ACells

WB method was used to detect apoptosis-related proteins. It was found that the proportion of Bcl-2/Bax in OGD/R + Butylphthalide group and OGD/R + miR-21 mimics group was significantly higher than that in OGD/R + mir-nc group, and lower than that in control group (Figures 3(a) and 3(b); *P* < 0.05). The proportion of caspase-3/GAPDH in these two groups was significantly lower than that in OGD/R + mir-NC group and higher than that in control group (Figures 3(a) and 3(c); *P* < 0.001), indicating that Butylphthalide treatment and overexpression of miR-21 could inhibit OGD/R-induced apoptosis.

### 3.4. Butylphthalide Exerts the Neuroprotective Effect through TLR4/NF-*κ*B Pathway

In order to clarify the specific mechanism of neuroprotective effect of Butylphthalide through miR-21, WB method was used to detect the expression of miR-21-related signaling pathway, TLR4/NF-*κ*B. The results showed that the p-TLR4/TLR4 level in OGD/R + Butylphthalide group and OGD/R + miR-21 mimics group was significantly lower than that in OGD/*R* + miR-NC group, and higher than that in control group. And the p-TLR4/TLR4 level in OGD/R + miR-NC group was higher than that in control group (Figures 4(a) and 4(b); *P* < 0.05). The level of p-NF-*κ*B/NF-*κ*B in OGD/R + Butylphthalide group and OGD/R + miR-21 mimics group was significantly decreased compared with that in OGD/R + miR-NC group (Figures 4(a) and 4(c); *P* < 0.001); the level of p-NF-*κ*B/NF-*κ*B in OGD/R + Butylphthalide group was similar to that in OGD/R + miR-21 mimics group and that in OGD/R + miR-NC group was higher than that in control group (Figures 4(a) and 4(c); *P* < 0.001).

## 4. Discussion

In this study, the possible mechanism of the neuroprotective effect of Butylphthalide was discussed. The previous study found that the level of miR-21 in the peripheral blood of ischemic stroke patients treated with butylphthalide was increased. In order to further clarify this phenomenon, the mouse model of a focal middle cerebral artery occlusion (MCAO) was established and it was found that the level of miR-21 in brain tissue of the mouse model of MCAO treated with Butylphthalide was significantly increased. What is more, Butylphthalide reduced the functional neurologic impairment score and infarct volume, showing neuroprotective effect. Studies have shown that its main mechanism is attributable to its anti-inflammatory and antiapoptotic properties [28, 29]. In addition, studies found that NBP can increase the local blood flow after cerebral ischemia, which may be beneficial for penumbral rescue [6]. It has been reported that NBP can reduce the activation of caspase-3 and caspase-9 and inhibit apoptosis after ischemic injury [19]. According to an in vitro study, NBP can protect cerebral microvascular endothelial cells from the injury induced by oxygen-glucose deprivation by upregulating the expression of Bcl-2 [30]. Another study found that NBP can reduce brain edema and downregulate RhoA expression, which is a downstream effector of RAS and can regulate the contraction of smooth muscle cells. The protective effect of NBP on endothelial cells and blood-brain barrier showed that NBP could recover the ischemic injury induced by angiotensin [31]. Fangfang Li et al. found that NBP treatment can reduce the volume of cerebral infarction 1 day after MCAO and significantly reduced the volume of cerebral infarction 3 days after MCAO [32]. In addition, Butylphthalide can also improve the functional neurologic impairment of mice. Butylphthalide can downregulate the expression of MMP-9, upregulate the expression of claudin-5, increase the expression of VEGF and GFAP, improve the ultrastructure of capillary endothelial cells of BBBs, and increase the expression of Nrf-2 and HO-1, having a protective effect on the brain of the mice [33]. In spontaneously hypertensive rats (SHR), NBP significantly reduced the functional neurologic impairment score and infarct volume and minimized the pathological changes of penumbra compared with placebo-treated control group [34]. All the above studies indicate that Butylphthalide plays a positive role in the neuroprotective effect of ischemic stroke, which also supports the results of this study. As the mechanism of action of Butylphthalide is diverse, further study is required.

RETRACTED

It should be noted that the level of miR-21 in the infarcted brain tissue was significantly decreased, and the level of miR-21 in the infarcted brain tissue of the mice in Butylphthalide-treated group was increased. Moreover, it was found that there was a negative correlation between the level of miR-21 and the neurological function score, indicating that miR-21 played an important role. Jiansuo Zhou et al. believed that the level of miR-21 in the plasma of patients with acute cerebral infarction was lower than that in control group. As the level of miR-21 was upregulated, the expression of Bcl-2 was upregulated. With the oxygen-glucose deprivation (OGD) model, it was found that miR-21 may have antiapoptosis effect in N2A neuroblastoma cells [35]. Separating the plasma exosomes of patients with ischemic stroke, Wang et al. found that the level of miR-21-5p in plasma exosomes of subacute patients and convalescents was significantly higher than that in control group, and the level of miR-21-5p and miR-30a-5p in hyperacute patients was significantly lower [36]. Therefore, the neuroprotective effect of butylphthalide may be based on the regulation of miR-21 level, thus affecting its targeted signaling pathway.

## 5. Conclusion

Further exploration was made on the specific mechanism of neuroprotective effect of Butylphthalide on MCAO by regulating miR-21. The experimental results showed that Butylphthalide could upregulate the survival rate of OGD/R cells, and the protective effect of upregulating the survival rate of Neuro2A cells was counteracted by inhibition of miR-21 expression with Butylphthalide treatment. Similarly, Butylphthalide treatment inhibited the production of reactive oxygen species and the cytotoxicity after OGD/R. However, inhibition of miR-21 expression significantly increased the cytotoxic reaction. In addition, it has been reported that ROS is involved in apoptosis [37]. Our results showed that Butylphthalide and miR-21 can inhibit caspase-3 and increase the proportion of Bcl-2/Bax, indicating that Butylphthalide can inhibit OGD/R-induced apoptosis through miR-21.

The expression of miR-21 can effectively inhibit TLR4/NF-*κ*B pathway, reducing the level of apoptosis and the release of inflammatory factors (25). We also found that Butylphthalide and miR-21 could inhibit p-TLR4/TLR4 and p-NF-*κ*B/NF-*κ*B in OGD/R model, which verified the effect of miR-21 on TLR4/NF-*κ*B in ischemic stroke. Butylphthalide may act on this pathway through miR-21, further affecting the apoptosis and activity of nerve cells to show its neuroprotective effect.

In conclusion, Butylphthalide has neuroprotective effect on the mouse model of MCAO. It may upregulate the level of miR-21 to inhibit neuronal apoptosis and ROS production and improve the proliferation activity. The specific mechanism may lie in inhibiting TLR4/NF-*κ*B pathway.

## Figures and Tables

**Figure 1:** Neuroprotective effect of Butylphthalide on cerebral ischemia model (mouse model of MCAO). (a) The functional neurologic impairment of the mice in MCAO model group was evaluated three days after reperfusion. The neurological function score of the mice in MCAO model group was significantly higher than that in MCAO + Butylphthalide-treated group. (b) 2,3,5-Triphenyltetrazolium chloride (TTC) was used to measure the volume of cerebral infarction. The volume of cerebral infarction of the mice in MCAO model group was larger than that in MCAO + Butylphthalide-treated group. (c) The volume of cerebral infarction of the mice in MCAO model group was significantly higher than that in MCAO + Butylphthalide-treated group. The volume of brain loss of the mice in MCAO model group was calculated three days after reperfusion. The brain loss of the mice in MCAO model group was significantly greater than that in MCAO + Butylphthalide-treated group. (d) qPCR method was used to detect the level of miR-21 in the brain tissue of the mice in MCAO group, MCAO + Butylphthalide-treated group, and sham group. It was found that the miR-21 level of the mice in MCAO group was the lowest, and that in Butylphthalide-treated group was higher than that in MCAO group. (e) The level of miR-21 in the brain tissue was negatively correlated with neurological impairment score.  ^*∗*^*P* < 0.05, ^*∗*^ ^*∗*^*P* < 0.01, ^*∗*^ ^*∗*^ ^*∗*^*P* < 0.001.

RETRACTED

**Figure 2:** Effects of Butylphthalide treatment and miR-21 overexpression on the proliferation of Neuro2Acells and ROS production. (a) qPCR method was used to detect the level of miR-21 in Neuro2A cells. The level of miR-21 in OGD/R + Butylphthalide group was significantly higher than that in OGD/R + Butylphthalide + miR-21 inhibitor group and control group. (b) MTT assay was used to detect the proliferation rate of Neuro2A. The proliferation rate of Neuro2A in OGD/R + Butylphthalide group was higher than that in OGD/R + Butylphthalide + miR-21 inhibitor group and control group, but there was no significant difference between OGD/R + Butylphthalide + miR-21 inhibitor group and control group. (c) Compared with OGD/R + Butylphthalide + miR-21 inhibitor group and OGD/R + miR-NC group, the ROS activity in OGD/R + Butylphthalide + miR-21 inhibitor group was significantly decreased, but there was no significant difference between OGD/R + Butylphthalide + miR-21 inhibitor group and OGD/R + miR-NC group.  ^*∗*^ ^*∗*^*P* < 0.01, ^*∗*^ ^*∗*^ ^*∗*^*P* < 0.001, ^*∗*^ ^*∗*^ ^*∗*^ ^*∗*^*P* < 0.0001.

**Figure 3:** Effects of Butylphthalide treatment and miR-21 overexpression on Neuro2A apoptosis. (a) The protein expression levels of Bcl-2, Bax, caspase-3, and GAPDH in OGD/R + Butylphthalide group, OGD/R + miR-21 mimics group, OGD/R + miR-NC group, and control group. (b) Statistical results showed that the proportion of Bcl-2/Bax in OGD/R + Butylphthalide group and OGD/R + miR-21 mimics group was significantly higher than that in OGD/R + miR-NC group, and the proportion of Bcl-2/Bax in OGD/R + miR-NC group was lower than that in control group. (c) Statistical results showed that the proportion of caspase-3/GAPDH in OGD/R + Butylphthalide group and OGD/R + miR-21 mimics group was significantly lower than that in OGD/R + miR-NC group, and the proportion of caspase-3/GAPDH in OGD/R + miR-NC group was higher than that in control group.  ^*∗*^*P* < 0.05, ^*∗*^ ^*∗*^*P* < 0.01, ^*∗*^ ^*∗*^ ^*∗*^*P* < 0.001, ^*∗*^ ^*∗*^ ^*∗*^ ^*∗*^*P* < 0.0001.

RETRACTED

**Figure 4:** Effects of Butylphthalide treatment and miR-21 overexpression on TLR4/NF-*κ*B of Neuro2A cells. (a) The protein expression levels of p-TLR4, p-TLR4, p-NF-*κ*B, and NF-*κ*B in OGD/R + Butylphthalide group, OGD/R + miR-21 mimics group, OGD/R + miR-NC group, and control group. (b) Statistical results showed that the proportion of p-TLR4/TLR4 in OGD/R + Butylphthalide group and OGD/R + miR-21 mimics group was significantly lower than that in OGD/R + miR-NC group, and the proportion of p-TLR4/TLR4x in OGD/R + miR-NC group was higher than that in control group. (c) Statistical results showed that the proportion of p-NF-*κ*B/NF-*κ*B in OGD/R + Butylphthalide group and OGD/R + miR-21 mimics group was significantly lower than that in OGD/R + miR-NC group, and the proportion of p-NF-*κ*B/NF-*κ*B in OGD/R + miR-NC group was higher than that in control group.  ^*∗*^*P* < 0.05, ^*∗*^ ^*∗*^*P* < 0.01, ^*∗*^ ^*∗*^ ^*∗*^*P* < 0.001, ^*∗*^ ^*∗*^ ^*∗*^ ^*∗*^*P* < 0.0001.

**Table 1:** The primer sequence of miR-21 and U6.

Gene	Forward (5′⟶3′)	Reverse (5′⟶3′)
miR-21	AGGCCCCTCTGAACCCTAAG3	CCAGAGGCATACAGGGACAAC3
U6	GCTTCGGCAGCACATATACTAAAAT	CGCTTCACGAATTTGCGTGTCAT3

## Data Availability

The datasets used and/or analyzed during the present study are available from the corresponding author on reasonable request.
